The article "miR-802 participates in the inflammatory process of inflammatory bowel disease by suppressing SOCS5" was retracted in 2024. Reasons: duplicated images; overlap with earlier publications; concerns about the data; concerns about the images.

#  miR-802 participates in the inflammatory process of inflammatory bowel disease by suppressing SOCS5

**DOI:** 10.1042/BSR20192257

**Published:** 2020-04-07

**Authors:** Jun Yao, Ruoyu Gao, Minghan Luo, Defeng Li, Liliangzi Guo, Zichao Yu, Feng Xiong, Cheng Wei, Benhua Wu, Zhenglei Xu, Dingguo Zhang, Jianyao Wang, Lisheng Wang

**Affiliations:** 1 Department of Gastroenterology, Jinan University of Second Clinical Medical Sciences, Shenzhen Municipal People’s Hospital, No. 1017, East Gate Road, Shenzhen City, Guangdong Province 518020, China; 2 Department of General Surgery, Shenzhen Children’s Hospital, No. 7019, Yitian Road Road, Shenzhen City, Guangdong Province 518026, China

**Keywords:** inflammatory bowel disease, mice colitis model, miR-802, SOCS5, Th17, TNF-α

## Abstract

The present study aims to reveal the detailed molecular mechanism of microRNA (miR)-802 in the progression of inflammatory bowel disease (IBD). IBD tissues were obtained from IBD patients, followed by CD4^+^ cells isolation. Then, qRT-PCR and ELISA were used to detect the expression of miR-802, suppressor of cytokine signaling 5 (SOCS5), interleukin (IL)-17A and tumor necrosis factor (TNF)-α. Transfection of miR-802 mimics and miR-802 inhibitor in CD4^+^ cells was detected by Western blot. TargetScan and luciferase reporter assay were used to detect the relationship between SOCS5 and miR-802. Finally, colitis mice model was established to verify whether miR-802 inhibitor was involved in the protective effect of colonic mucosa. The miR-802 was highly expressed in inflamed mucosa and PBMC cells of IBD. The highest expression of miR-802 was observed in CD4^+^ T cells based on different immune cell subsets analysis. SOCS5 was the target gene of miR-802. The mice model experiments showed that blockade of miR-802 could alleviate mice colitis. Our study suggests that up-regulation of miR-802 plays an important role in inflammatory process of IBD via targeting SOCS5. Moreover, the differentiation of Th17 and secretion of TNF-α in IBD could be stimulated by miR-802.

## Introduction

Inflammatory bowel disease (IBD), with two major subtypes including ulcerative colitis (UC) and Crohn’s disease (CD), is typically chronic and easy to relapse [1]. In recent years, the morbidity and mortality of IBD is increasing worldwide [2,3]. IBD is commonly known to be caused by over-reacted immune responses against internal or external microbes or antigens. However, the detailed pathogenesis is unclear.

T cells including effector T cells, regulatory T cells and T helper 17 (Th17) cells have been proved to play important roles in IBD [1]. Herein, Th17 cells are participated in the development of IBD and have potentials to be used as therapeutic target for IBD [4]. Th17 cells regulate the secretion of many kinds of cytokines including tumor necrosis factor α (TNF-α) [5,6]. Furthermore, the expression level of TNF-α is proved to be associated with the process of IBD [7]. Therefore, the TNF-α antagonists represent a useful therapy against IBD [8].

The article "miR-802 participates in the inflammatory process of inflammatory bowel disease by suppressing SOCS5" was retracted in 2024. Reasons: duplicated images; overlap with earlier publications; concerns about the data; concerns about the images.

The microRNA (miRNA) is demonstrated to be participated in Th1/Th17 responses in IBD [9]. Commonly, several miRNAs affect the biological function of T cells or the expression of cytokines by targeting certain genes such as suppressor of cytokine signaling 5 (SOCS5) [10]. For example, a previous study indicated that T-cell differentiation is controlled by miR-124-mediated suppression of SOCS5 [11]. miR-301a can regulate Th17 responses and TNF-α expression during the development of IBD [12]. However, the detailed mechanism of miR-802 in IBD is unclear.

In the present study, CD4^+^ cells obtained from IBD patients were subjected to series of analyses via transfection of miR-802 mimics or inhibitors to uncover the biological functions of miR-802. Furthermore, the 2,4,6-trinitrobenzenesulfonic acid (TNBS)-induced colitis mice model was established to investigate whether miR-802 inhibitor had protective effects of colonic mucosa. Based on the experiments above, the present study proposed to understand the molecular mechanism of miR-802 in the progression of IBD.

## Methods

### Patients and control subjects

From June 2016 to August 2018, a total of 100 IBD patients were selected from Department of Gastroenterology in our hospital. Based on the diagnostic criteria published by the American College of Gastroenterology (ACG) in 2010, 50 patients were diagnosed as CD, of which 30 were active CD (A-CD) and 20 were remission CD (R-CD); another 50 patients were diagnosed as UC, of which28 were active UC (A-UC) and 22 were remission UC (R-UC), [13]. Meanwhile, a total of 20 healthy volunteers from the Physical Examination Center of our hospital (from January 2017 to January 2018) were selected as healthy control (HC) group. Written informed consent was obtained from all patients and healthy volunteers prior to the study. The present study was approved by the Ethics Committee of our hospital (ethic vote 36/40). The clinical information of all the patients was shown in Table 1.

**Table 1:** The detail clinical information of all the subjects

	HC	CD (A/R)	UC (A/R)	*P*
Number	20	50 (30/20)	50 (28/22)	–
Age	35 ± 8.1	32.8 ± 7.3	35.1 ± 6.45	0.54
Gender				
Male	11	27 (15/12)	21(14/7)	0.71
Female	9	23 (15/8)	29 (16/13)	
Disease duration (months)		45 ± 10	43 ± 8.45	0.41
Mayo scores (UC)			7.89 ± 1.56/1.2 ± 0.69	
CDAI (CD)		170 ± 30/70 ± 11		
Disease extent (UC)				
E1			8 (6/2)	
E2			20 (12/8)	
E3			22 (11/11)	
Disease location (CD)				
L1		8 (4/4)		
L2		16 (10/6)		
L3		26(16/10)		
L4		0		
CRP (mg/l)	38 ± 9.6	35 ± 7.9		0.16

Abbreviations: CD, Crohn’s disease; CDAI, Crohn’s disease activity index; CRP, C-reactive protein; HC, healthy control; UC, ulcerative colitis.

The article "miR-802 participates in the inflammatory process of inflammatory bowel disease by suppressing SOCS5" was retracted in 2024. Reasons: duplicated images; overlap with earlier publications; concerns about the data; concerns about the images.

The intestinal mucosa tissues obtained from all participants were cutted into square (0.5 cm × 0.5 cm). Then, the intestinal epithelial cells (IEC) in the tissues were removed by treating with 2 mM DTT and 1 mM EDTA in PBS for 30 min, at 37°C. Next, the tissues were digested by 2% FBS-RPMI-Collagenase A (1 mg/ml, Roche, Mannheim) for 40 min at 37°C. Then, the digested cells were harvested by density gradient centrifugation using 40% and 70% Percoll-RPMI solutions.

A total of 10 ml peripheral blood was obtained from each participant. Then, the human mononuclear cells (PBMCs) were isolated from the peripheral blood samples by Ficoll-Paque density gradient centrifugation (GE Healthcare Biosciences). Next, the PBMCs were cultured in RPMI1640 medium (Hyclone) with 10% FBS (Hyclone) in a saturated humidity incubator (MCO-15AC, SANYO, Japan) at 37°C with 5% CO_2_. Then, the CD4^+^ T cells, CD8^+^ T cells, B cells and monocytes were separated from the PBMCs using a Magnetic Cell Sorting System (Invitrogen Dynal AS, Oslo, Norway) in accordance with the manufacturer’s instructions.

### Real-time quantitative PCR

Total RNAs were extracted from the sample of each participants and quantified using TRIzol reagent (invitrogen, San Diego, U.S.A.), and reverse-transcribed using FastQuant RT Kit (Tiangen, Beijing, China) in accordance with the manufacturers’ instructions. The RT-qPCR was performed on ABI PRISMR 7300 Sequence Detection System (Applied Biosystems, Foster City, CA, U.S.A.). The β-actin served as internal control. The sequences for all primers were shown in Table 2. The reaction conditions were as follows: 95°C for 3 min, 40 cycles at 95°C for 10 s, 60°C for 30 s and 72°C for 20 s. Fluorescence signals were collected at the end point of each cycle extension, followed by the amplification curve investigation. Relative expression of candidate genes were calculated using 2^−∆∆CT^ method [14].

**Table 2:** Amplified sequences of genes and their primers

Primer	Sequence
miR-802	Forward:5′-ACGTTGTGTAGCTTATCAGACTG -3′
	Reverse: 5′- AATGGTTGTTCTCCACACTCTC -3′
U6	Forward: 5′-CTCGCTTCGGCAGCACA-3′
	Reverse: 5′-AACGCTTCACGAATTTGCGT-3′
IL-17A	Forward: 5′-ACTCCTGGGAAGACCTCATTG -3′
	Reverse: 5′-GGCCACATGGTGGACAATCG-3′
RORC	Forward: 5′-CAATGGAAGTGGTGCTGGTTAG-3′
	Reverse: 5′- GGGAGTGGGACAAGTCAAAGAT-3′
TNF-α	Forward: 5′-GGTCCCCAAAGGGATGAGAAGT-3′
	Reverse: 5′-CCACTTGGTGGTTTGCTACGACG-3′
SOCS5	Forward: 5′-TGGAACAATAGCGGATAGAGC-3′
	Reverse: 5′-TTGCCTCACTCAAATACCACA-3′
β-actin	Forward: 5′-ACACCTTCTACAATGAGCTG-3′
	Reverse: 5′-CTGCTTGCTGATCCACATCT-3′
Si-SOCS5	Forwrad:5′- AAACATTTTAAAATT AACTTTT-3′
	Reverse:5′- TGTAAATATCTTTCAATTTGTTTT -3
siNC	Forwrad:5′-UUCUCCGAACGUGUCACGUTT-3′
	Reverse:5′-ACGUGACACGUUCGGAGAATT-3′

Abbreviations: IL-17A, interleukin 17A; NC, normal control; RORC, RAR related orphan receptor C; SOCS5, suppressor of cytokine signaling 5.

The article "miR-802 participates in the inflammatory process of inflammatory bowel disease by suppressing SOCS5" was retracted in 2024. Reasons: duplicated images; overlap with earlier publications; concerns about the data; concerns about the images.

### Cell transfection

The CD4^+^ T cells in logarithmic phase were seeded in 6-well plates at a density of 6 × 10^5^ cells per well, followed by incubating at 37°C with 5% CO_2_ until reaching 60% confluency. Then, miR-802 mimics, miR-802 inhibitor, mimics-negative control (mimics-NC) or inhibitor-NC (Shanghai Genepharma Co., Ltd.) were respectively added and co-incubated in RPMI1640 medium. Therefore, five groups were divided into Mock group, mimics-NC group, miR-802 mimics group, inhibitor-NC group and miR-802 inhibitor group.

Silencing of SOCS5 gene was realized by RNA interference technology. All siRNAs were synthesized by Shanghai Sagon bio-Tec Co., Ltd (Shanghai, China). Based on different transfection with si-NC, si-SOCS5, miR-802 inhibitor and inhibitor-NC, cells were divided into si-NC + inhibitor-NC group, si-NC + miR-802 inhibitor group, si-SOCS5 + inhibitor-NC group and si-SOCS5 + miR-802 inhibitor group.

### Luciferase reporter assay

The potential reactions between SOCS5 and miR-802 were predicted by TargetScan (http://targetscan.org/). Based on the prediction, a wild-type (SOCS5-WT) and mutant (SOCS5-MUT) 3′UTR fragment of the SOCS5 were synthesized. Then, the SOCS5-WT and SOCS5-MUT were cloned into the PsiCHECK-2 vector (Promega, Madison, WI, U.S.A.), respectively. After inoculation in 24-well plates (5 × 10^5^/well) for 24 h, miR-802 mimic or miR-802 NC, SOCS5-WT and SOCS5-MUTwere co-transfected into HEK-293T by Lipofectamine 3000 (Thermo Fisher Scientific), followed by measuring by Dual Luciferase Reporter Assay Kit (Promega, E1910, WI, U.S.A.) 48 h after transfection.

### Western blot

After transfection, the cells were lysed by RIPA lysis buffer. Then, the extracted proteins were quantified using bicinchoninic acid (BCA) kit (Thermo Fisher Scientific, Runcorn, Cheshire, U.K.). Next, the proteins were separated by 10% SDS-PAGE gels, and then transferred onto polyvinylidenefluoride (PVDF) membranes. After being blocked with 5% skim milk, the membrane was incubated with primary antibodies including rabbit anti-human GAPDH (1:1000, ab9485, Abcam) or SOCS5 (1:1000, ab97283, Abcam) at 4°C overnight, respectively. Herein, GAPDH was used as internal control. Then, the membrane was incubated with secondary antibodies (goat anti-rabbit IgG, 1:10,000, Sigma Company) at room temperature for 1 h. Finally, the membrane was visualized by staining with diaminobenzidine (DAB).

The article "miR-802 participates in the inflammatory process of inflammatory bowel disease by suppressing SOCS5" was retracted in 2024. Reasons: duplicated images; overlap with earlier publications; concerns about the data; concerns about the images.

### ELISA

The expression levels of IL-17A and TNF-α were determined by ELISA kits (R&D Systems, U.S.A.) according to manufacturer’s instructions. Optical density (OD) values at 450/550 nm were measured by the microplate reader (sPectraMAX 340, Molecular Devices, Sunnyvale, CA, U.S.A.). The standard was drawn, and the concentration of the samples was calculated according to the standard curve.

### TNBS-induced colitis model construction

A total of 24 female BALB/c mice (8–10 weeks) were purchased from the Experimental Animal Center of Academy of Sciences (Shanghai, China), and randomly divided into TNBS group (*n* = 12) and control group (*n* = 12). All mice were subjected to anesthesia with sodium pentobarbital (0.05 mg/g, Chuangdong Co., Chongqing, China) and polyethylene catheter. Then, a total of 2.0–2.5 mg of TNBS (dissolved in 50% ethanol) was administrated to each mice in TNBS group via enteroclysis (the depth of anal intubation was 5 cm), followed by heading down the mice for at least 10 min. Meanwhile, the mice in control group were treated with equal volume of 50% ethanol. Next, the mice in TNBS group were intracolonicaly administered with three optical density (OD) dose of inhibitor-NC and miR-802 inhibitor for four consecutive days. Then, after all mice were executed via brokening neck, the colon tissues were obtained, fixed with 10% paraformaldehyde, embedded with paraffin, sliced, and stained with hematoxylin and eosin (HE). The present study was approved by the ethics committee of Jinan University of Second Clinical Medical Sciences, Shenzhen Municipal People’s Hospital, and all experiments were in accordance with the guide for the care and use of laboratory animals established by United States National Institutes of Health (Bethesda, MD, U.S.A). All the animal experiments were conducted in the Science and Education Building of Jinan University of Second Clinical Medical Sciences, Shenzhen Municipal People’s Hospital.

### Flow cytometry

The digested cells of colonic mucosa were stimulated with PMA (50 ng/ml, eBioscience) and ionomycin (750 ng/ml, eBioscience) for 3 h. Then, brefeldin A (3 μg/ml, eBioscience) was added to the medium and incubated for another 2 h. Next, the cells were incubated with FITC-labeled anti-CD4 antibody at 4°C for 30 min. After permeabilization, PE-labeled anti-IL-17A was added into the cells, followed by another incubation for 20 min in dark. The dyed cells were analyzed by flow cytometry (FACS Calibur, BD Biosciences, San Jose, CA, U.S.A.).

The article "miR-802 participates in the inflammatory process of inflammatory bowel disease by suppressing SOCS5" was retracted in 2024. Reasons: duplicated images; overlap with earlier publications; concerns about the data; concerns about the images.

### Statistical analysis

SPSS 22.0 (Chicago, IL, U.S.A.) and GraphPad Prism 7.01 were used for data analyses in this study. All data were represented as the mean ± standard deviation (SD). Significant differences between two groups were assessed using Student’s *t* test, while one-way ANOVA was used for more than two groups. Tukey’s multiple comparison test was used for the pairwise comparison after ANOVA. *P* < 0.05 was considered as statistically significance.

## Results

### The miR-802 was up-regulated in colonic mucosa and PBMC cells of IBD

The miR-802 expression was assessed by RT-qPCR in colonic mucosa of human patients or healthy controls (HC). The results showed that miR-802 was significantly increased in both A-CD group and A-UC group compared with that in HC group (*P* < 0.05, Figure 1A). Similarly, miR-802 was highly expressed in PBMC of both A-CD group and A-UC group compared with HC group (*P* < 0.05, Figure 1B). The expression levels of miR-802 in the inflammatory mucosa of the same A-CD or A-UC patients were higher than that in the non-inflammatory mucosa (*P* < 0.05; Figure 1C,D).

**Figure 1:** The expression of microRNA-802 in inflammatory bowel disease inflamed mucosa and peripheral blood mononuclear cells (**A**) The RT-qPCR detection of miR-802 expression in colonic mucosa of healthy control (HC) (*n* =20) and IBD group (A-CD, *n* = 30; R-CD, *n* = 20; A-UC, *n*=28; R-UC, *n*=22); ***, *P*<0.001. (**B**) The expression of miR-802 in PBMC of HC and IBD patients detected by RT-qPCR; ***, *P* < 0.001. (**C** and **D**) The expression of miR-802 in inflammatory and non-inflammatory mucosa of the same patient with active ulcerative colitis or active Crohn’ disease (*n* = 30); ***, nn*P* < 0.001. (**E**) The expression of miR-802 in peripheral blood CD4^+^, CD8^+^ T cells, B cells, monocytes and monocyte-derived-dendritic-cells (MDDC) of eight healthy volunteers; ***, *P* < 0.001 when compared with B cells. (**F**) The expression of miR-802 in IEC, CD4^+^, CD8^+^ T cells and B cells separated from normal tissues (*n* = 8). ***, *P* < 0.001 when compared with B cells. One-way ANOVA was used for the present study. Tukey’s multiple comparison test was used for the pairwise comparison after ANOVA.

### The miR-802 promoted Th17 differentiation and TNF-α secretion

First, to investigate the expression of miR-802 in different immune cell subsets, CD4^+^, CD8^+^ T cells, B cells and monocytes in peripheral blood were prepared from eight healthy volunteers. The results of RT-qPCR analysis showed that the highest expression of miR-802 was found in CD4^+^ T cells (*P* < 0.05, Figure 1E) of peripheral blood. In mucosa, the expression of miR-802 in IEC and CD4 + T cells was significantly higher than that in CD8^+^ T cells and B cells (*P* < 0.05, Figure 1F). Furthermore, the role of miR-802 in different lineages of CD4^+^ T cells was investigated in HC group (Figure 2A). The results showed that the expression of miR-802 was highest in Th17 cells, and the expression of miR-802 in Treg cells was significantly decreased compared with that in Th0 cells. Moreover, to reveal whether miR-802 was involved in Th17 cell differentiation, the miR-802 mimics and miR-802 were into CD4^+^ T cells (Figure 2B). The results showed that the relative expression of miR-802 in miR-802 mimics group was significantly higher than that in mimics-NC group (*P* < 0.05). Meanwhile, the relative expression of miR-802 in miR-802 inhibitor group was significantly lower than that in inhibitor-NC group (*P* < 0.05). Furthermore, the proportion of IL-17A^+^ cells in miR-802 mimics group was significantly higher than that in mimics-NC group (*P* < 0.05), while the proportion of IL-17A^+^ cells in the miR-802 inhibitor group was significantly lower than that in the inhibitor-NC group (*P* < 0.05, Figure 2C), indicating that miR-802 promoted the cell differentiation of Th17 cells.

The article "miR-802 participates in the inflammatory process of inflammatory bowel disease by suppressing SOCS5" was retracted in 2024. Reasons: duplicated images; overlap with earlier publications; concerns about the data; concerns about the images.

**Figure 2:** The microRNA-802 promoted Th17 differentiation and TNF-α secretion in inflammatory bowel disease (**A**) CD4^+^ cells of healthy control (HC) cultured in polarized culture for 5 days; the expression of miRNA-802 in Th1, Th2, Th17 and Treg cells was detected by qRT-PCR; CD4^+^ T cells cultured with anti-CD3/CD28 alone were defined as Th0 cells to serve as controls. (**B**) Transfection efficiency. (**C**) Differentiation of Th17 cells detected by flow cytometry. (**D–F**) The expression of IL-17A, TNF-α and RORC detected by qRT-PCR. (**G** and **H**) The expression of IL-17A and TNF-α detected by ELISA. *P < 0.05. One-way ANOVA was used for the present study. Tukey’s multiple comparison test was used for the pairwise comparison after ANOVA.

Furthermore, ELISA and RT-qPCR were performed to reveal the effect of miR-802 on Th17 differentiation and immune function in CD4^+^ T cells isolated from IBD patients (Figure 2D–H). The results showed that both transcription and protein expression levels of IL-17A and TNF-α in miR-802 mimics group were significantly higher than those in other groups, regardless of whether CD4^+^ T cells were generated from HC, CD or UC patients (*P* < 0.05). At the same time, miR-802 mimics significantly promoted the expression of Th17 cell-specific transcription factor RORC. Reversely, miR-802 inhibitor inhibited the expression of RORC (*P* < 0.05).

The article "miR-802 participates in the inflammatory process of inflammatory bowel disease by suppressing SOCS5" was retracted in 2024. Reasons: duplicated images; overlap with earlier publications; concerns about the data; concerns about the images.

### SOCS5 was the target gene of miR-802

By Targetscan prediction, the binding site of miR-802 to SOCS5 was the 3′-UTR region, SOCS5 WT and SOCS5 mutant referred to wild-type and mutant 3′UTR sequences recognized by mature miR-802, respectively (Figure 3D). The results of the RT-qPCR analysis showed that SOCS5 was low expressed in tissues (Figure 3B,C) and PBMCs (Figure 3D) in IBD patients, while the expression level of miR-802 was negatively correlated with that of SOCS5. The results of luciferase reporter assay showed that in HEK-293T cells, the luciferase activity decreased significantly in the both miR-802 mimics group and SOCS5 wild-type recombinant vector transfection group (*P* < 0.05, Figure 3E). Moreover, expression of SOCS5 in CD4^+^ T cells in each treatment group was assessed to determine if miR-802 suppressed expression of SOCS5, leading to negative correlation between expression of miR-802 and SOCS5 mRNA (Figure 3F). The results showed that the expression level of SOCS5 was significantly decreased in the miR-802 mimics group and increased in miR-802 inhibitor group (*P* < 0.05).

**Figure 3:** SOCS5 was the target gene of micro-RNA802 (**A**) Targetscan predicted the target binding sites between SOCS5 and miR-802. (**B**) RT-qPCR was used to detect the expression of SOCS5 in colon mucosa of healthy control (HC) and IBD patients; ***, *P* < 0.001. (**C**) Correlation analysis between miR-802 and SOCS5. (**D**) RT-qPCR was used to detect the expression of SOCS5 in PBMC of HC and IBD patients; ***, *P* < 0.001. (**E**) The results of luciferase reporter gene activity detection; *, *P* < 0.05. (**F**) The RT-qPCR was used to detect the expression of SOCS5 in CD4^+^ cells after transfection. *, *P* < 0.05. One-way ANOVA was used for the present study. Tukey’s multiple comparison test was used for the pairwise comparison after ANOVA.

### SOCS5 eliminated the effect of miR-802 on CD4^+^ cells

The results of RT-qRCR showed that the expression of SOCS5 in si-SOCS5 group was significantly lower than that in si-NC group (*P* < 0.05, Figure 4A). Compared with the si-NC + inhibitor-NC group, the expression of IL-17A, TNF-alpha and RORC in the si-SOCS5 + inhibitor-NC group were significantly increased and in si-NC + miR-802 inhibitor group were significantly decreased (*P* < 0.05, Figure 4B–F). Meanwhile, there was no significant difference of Th17 differentiation and TNF-α expression level between si-SOCS5 + miR-802 inhibitor group and si-NC + inhibitor-NC group (*P* > 0.05).

**Figure 4:** SOCS5 eliminated the effect of micro-RNA802 on CD4+ cells (**A**) Detection of interference efficiency by qRT-PCR. (**B–D**) The interaction between miR-802 and SOCS5 on the mRNA expression level of IL-17A, TNF-a and RORC. (**E–F**) The interaction between miR-802 and SOCS5 on the protein expression level of IL-17A and TNF-α. *, *P* < 0.05 when compared with the si-NC + inhibitor-NC group; #, *P* < 0.05 when compared with the si-SOCS5 + inhibitor-NC group; &, *P* < 0.05 when compared with the si-NC+miR-802 inhibitor group. One-way ANOVA was used for the present study. Tukey’s multiple comparison test was used for the pairwise comparison after ANOVA.

The article "miR-802 participates in the inflammatory process of inflammatory bowel disease by suppressing SOCS5" was retracted in 2024. Reasons: duplicated images; overlap with earlier publications; concerns about the data; concerns about the images.

### Effect of miR-802 blocking on TNBS-induced colitis in mice

**Figure 5:** Effect of micro-RNA802 blockade on TNBS-induced colitis in mice (**A**) The RT-qPCR was used to detect the expression of miR-802 in mouse colonic mucosa; *, *P* < 0.05. (**B** and **C**) The RT-qPCR and Western blot were used to detect the expression of SOCS5 in colonic mucosa of mice; *, *P* < 0.05. (**D**) The percentage of current and original body weight over a period of time; *, *P* < 0.05 when compared with control group; #, *P* < 0.05 when compared with TNBS + inhibitor-NC group. (**E**) The changes of disease activity index; *, *P* < 0.05 when compared with control group; #, *P* < 0.05 when compared with TNBS + inhibitor-NC group. (**F**) Colon length; *, *P* < 0.05. (**G**) HE staining (original magnification ×200) and pathological score; *, *P* < 0.05. One-way ANOVA was used for the present study. Tukey’s multiple comparison test was used for the pairwise comparison after ANOVA.

The results of RT-qPCR and Western blot (Figure 5A–C) showed that the expression of miR-802 was significantly increased and SOCS5 was decreased in TNBS group compared with that in the control group (*P* < 0.05). The expression of miR-802 was significantly decreased and SOCS5 was increased in TNBS + miR-802 inhibitor group compared with that in TNBS group (*P* < 0.05). Moreover, the body weight of mice was significantly decreased and the DAI index of mice was increased in TNBS group compared with that in control group (*P* < 0.05). Meanwhile, the body weight of mice was significantly increased and the colon length of mice was decreased in TNBS + miR-802 inhibitor group compared with that in TNBS group (*P* < 0.05, Figure 5D–F). Furthermore, the results of HE staining showed that the monocytes were seriously infiltrated in TNBS group and TNBS + inhibitor-NC group compared with that in control group. Meanwhile, the monocyte infiltration and inflammation were significantly reduced in TNBS + miR-802 inhibitor group compared with that in control group (Figure 5G).

### miR-802 blocking inhibited Th17 differentiation and TNF-α secretion

The results of flow cytometry and RT-qPCR analysis showed that the proportion of IL-17A^+^ cells were significantly increased, and the expression levels of IL-17A, RORC and TNF-α were significantly increased in the TNBS group compared with that in control group (*P* < 0.05, Figure 6A–D). The percentage of IL-17A^+^ cells as well as expression of IL-17A, RORC and TNF-α were significantly decreased in the TNBS + inhibitor-NC group compared with that in TNBS + miR-802 inhibitor group (*P* < 0.05).

The article "miR-802 participates in the inflammatory process of inflammatory bowel disease by suppressing SOCS5" was retracted in 2024. Reasons: duplicated images; overlap with earlier publications; concerns about the data; concerns about the images.

**Figure 6:** Blockade of micro-RNA802 inhibited Th17 differentiation and TNF-α secretion (**A**) Th17 differentiation detected by flow cytometry. (**B–D**) The expression of IL-17A, RORC and TNF-α detected by RT-qPCR. One-way ANOVA was used for the present study. Tukey’s multiple comparison test was used for the pairwise comparison after ANOVA. The experiments were repeated for three times.

## Discussion

CD4^+^ T cells in PBMCs can induce the production of interleukins in inflammation process of inflammatory diseases such as IBD [15]. During this process, miRNAs contribute to the regulation of CD4^+^ T cells in the development of disease [16]. The blood miRNAs expression analysis is successfully used to reveal inflammation associated biomarkers in patients with IBD [17]. A previous study showed that miRNA-146a was associated with the differentiation of CD4^+^ T cells [18]. Chen et al. indicated that miRNA-155 was up-regulated in CD4^+^ T cells of TNBS-induced colitis [19].

The miR-802 expression has been studied in human diseases and mice models [20]. A previous study showed that the up-regulation of miR-802 stimulated cell cycle progression [21]. As a proinflammatory mediator that participates in inflammatory responses, human angiotensin II receptor is proved to be regulated by miR-802 in intestinal epithelial cells [22].

Actually, the biological function of miRNAs in inflammatory process are commonly realized by targeting certain genes [23]. During this process, the relation between miRNAs (such as miR-432) and SOCS family (such as SOCS5) has been revealed [24]. A previous study indicated that the suppression of miR-221 promoted neuropathic pain via targeting SOCS1 [25]. Meanwhile, the T-cell differentiation is proved to be realized by controlling miR-124 mediated suppression on SOCS5 [11]. In the present study, the RT-qPCR analysis showed that the miR-802 was up-regulated in both tissues and PBMCs of IBD patients. The high expression of miR-802 was observed in CD4^+^ T cells. Meanwhile, as the target gene of mir-802 that investigated by TargetScan, SOCS5 eliminated the effect of miR-802 on CD4^+^ cells. Thus, based on these results, we speculated that the overexpression of miR-802 might take part in the inflammatory process in IBD by suppressing SOCS5.

The article "miR-802 participates in the inflammatory process of inflammatory bowel disease by suppressing SOCS5" was retracted in 2024. Reasons: duplicated images; overlap with earlier publications; concerns about the data; concerns about the images.

Th17 and TNF-α are important factors for mediating inflammation during the development of inflammatory disease [26,27]. TNF-α contributes to the development of asthma by promoting Th17 expression during immune responses [28]. A previous study showed that Th17 and TNF-α in the cells of bone marrow can lead to osteoclast differentiation and bone destruction in IBD [29]. Th17 cells are proved to be associated with the development of IBD [4]. Inhibiting Th17-associated cytokine is a novel breakthrough for clinical treatment of IBD [30,31]. During this process, miRNA is proved to be participated in the regulation of Th17 and TNF-α in disease [9]. Li et al. proved that miR-181a regulated adipogenesis by targeting TNF-α in the porcine model [32]. Although the correlation between miRNA-802 and TNF-α has been mentioned in PBMCs of IBD in previous study [33], the specific effects of miR-802 on Th17 and TNF-α in IBD is still unclear. In the present study, the ELISA and qRT-PCR results showed that the transcription and protein levels of IL-17A and TNF-α were significantly increased in the miR-802 mimics group. Meanwhile, the mice model experiments showed that blocking of miR-802 could alleviate mice colitis.

In conclusion, miR-802 takes part in the inflammatory process of IBD via suppressing SOCS5. Moreover, miR-802 promotes Th17 differentiation and TNF-α secretion in IBD. Furthermore, miR-802 inhibitor protected the function of intestinal mucosa, and might be novel breakthrough for clinical treatment of IBD.

## Abbreviations

CD: Crohn’s disease
CDAI: Crohn’s disease activity index
CRP: C-reactive protein
IBD: inflammatory bowel disease
IL: interleukin
miR: microRNA
SOCS5: suppressor of cytokine signaling 5
TNF: tumor necrosis factor
